# The Role and Mechanism of SIRT6 in Regulating Phenotype Transformation of Vascular Smooth Muscle Cells in Abdominal Aortic Aneurysm

**DOI:** 10.1155/2022/3200798

**Published:** 2022-01-06

**Authors:** Xiaomei Guan, Hai Xin, Meiling Xu, Jianlei Ji, Jun Li

**Affiliations:** ^1^Department of Vascular Surgery, Affiliated Hospital of Qingdao University, Qingdao 266700, China; ^2^Department of Interventional Operating Room, Affiliated Hospital of Qingdao University, Qingdao 266700, China; ^3^Department of Kidney Transplantation, Affiliated Hospital of Qingdao University, Qingdao 266700, China

## Abstract

**Background:**

Data mining of current gene expression databases has not been previously performed to determine whether sirtuin 6 (SIRT6) expression participates in the pathological process of abdominal aortic aneurysm (AAA). The present study was aimed at investigating the role and mechanism of SIRT6 in regulating phenotype transformation of vascular smooth muscle cells (VSMC) in AAA.

**Methods:**

Three gene expression microarray datasets of AAA patients in the Gene Expression Omnibus (GEO) database and one dataset of SIRT6-knockout (KO) mice were selected, and the differentially expressed genes (DEGs) were identified using GEO2R. Furthermore, Gene Ontology (GO) and Kyoto Encyclopedia of Genes and Genomes (KEGG) analyses of both the AAA-related DEGs and the SIRT6-related DEGs were conducted.

**Results:**

GEO2R analysis showed that the expression of SIRT6 was downregulated for three groups and upregulated for one group in the three datasets, and none of them satisfied statistical significance. There were top 5 DEGs (KYNU, NPTX2, SCRG1, GRK5, and RGS5) in both of the human AAA group and SIRT6-KO mouse group. Top 25 ontology of the SIRT6-KO-related DEGs showed that several pathways including tryptophan catabolic process to kynurenine and negative regulation of cell growth were enriched in the tissues of thickness aortic wall biopsies of AAA patients.

**Conclusions:**

Although SIRT6 mRNA level itself did not change among AAA patients, SIRT6 may play an important role in regulating several signaling pathways with significant association with AAA, suggesting that SIRT6 mRNA upregulation is a protective factor for VSMC against AAA.

## 1. Background

Abdominal aortic aneurysm (AAA) usually refers to the abdominal aorta with tumor-like expansion, and the maximum cross-sectional diameter of the abdominal aorta exceeds 3 cm, or the diameter of the abdominal aorta is 1.5 times or more than the diameter of the adjacent normal artery [1]. Previous studies have shown that the mortality rate after AAA rupture is as high as 80% [2]. According to statistics, the annual death toll caused by AAA rupture in the United States reaches 15,000 [3]. Therefore, the occurrence, development, and rupture of AAA are the critical challenges related to public health.

Vascular smooth muscle cells (VSMCs) are the main cell components of the blood vessel wall, which play an important role in maintaining vascular structure and remodeling under the stimulation in the surrounding environment. The main initiating factor of aortic aneurysm formation is the transformation of VSMCs from the physiological contraction phenotype (differentiation) to pathological synthesis and inflammatory state [4, 5]. This process involves the coordinated downregulation of smooth muscle contraction gene expression and contractility, as well as the production of matrix metalloproteinases (MMPs) and proteoglycans, leading to the degradation of the extracellular matrix, weakening of the aortic wall, and eventually rupture [6, 7]. Smooth muscle cell (SMC) contractile elements, such as smooth muscle actin (a-SMA) [8], myosin light-chain kinase (MLCK) [9, 10], and smooth muscle myosin heavy chain 11 (SMMHC11) [11, 12], and other gene mutations are related to the occurrence and development of AAA, and it has been found that it may trigger the phenotypic transformation of SMC. Nevertheless, most of AAA are sporadic with no obvious genetic characteristics [13]. The genes and signal pathways related to sporadic nonsyndromic AAA are still unclear. In addition, it is still unclear which link the contractile phenotype SMC transforms to the synthetic phenotype SMC.

The sirtuin family is a group of class III histone deacetylases that catalyze the deacetylation of histone and nonhistone lysine residues. The sirtuin family plays an important role in regulating aging and energy metabolism [14]. Sirtuin 6 (SIRT6), a member of the sirtuin family, is located in the nucleus and has both deacetylase activity and ADP-ribosyltransferase activity [15]. SIRT6, located on human chromosome 19, includes three important functional regions: the core catalytic region, the C-terminal nuclear localization signal region, and the N-terminal histone deacetylase functional region [16]. Studies have shown that SIRT6 can delay the occurrence and development of atherosclerosis by reducing endothelial cell damage, inhibiting inflammation and oxidative stress, regulating the balance of glucose and lipid metabolism, reducing foam cells, and stabilizing atherosclerosis [17]. Grootaert et al. also demonstrated that SIRT6 protein expression was reduced in human and mouse plaque VSMCs and that its overexpression protected VSMCs and inhibited the development of atherosclerosis [18]. However, there are currently few studies on whether SIRT6 also plays an important role in AAA. Therefore, in the present study, four microarray datasets from the Gene Expression Omnibus (GEO) database were used to identify differentially expressed genes (DEGs) in AAA and SIRT6-knockout (KO) mice. Subsequently, the potential molecular mechanisms of SIRT6 involvement in the pathological process of AAA were assessed by Gene Ontology (GO) annotation and Kyoto Encyclopedia of Genes and Genomes (KEGG) pathway enrichment analysis.

## 2. Material and Methods

### 2.1. Expression Database of the AAA Groups

The gene expression profile data for AAA tissue were downloaded from the GEO database (https://www.ncbi.nlm.nih.gov/gds). The GEO accession numbers are GSE57691 [19], GSE7084 [20], and GSE47472. GSE57691 with the GPL10558 platform (Illumina HumanHT-12 V4.0 expression beadchip) was obtained from 20 patients with small AAA (mean maximum aortic diameter = 54.3 ± 2.3 mm) and 29 patients with large AAA (mean maximum aortic diameter = 68.4 ± 14.3 mm), and the relative aortic gene expression was compared with that of 10 control aortic specimens of organ donors. GSE7084 was based on the GPL570 platform (Affymetrix Human Genome U133 Plus 2.0 Array) and GPL2507 platform (Sentrix Human-6 Expression BeadChip) and was obtained from either autopsy within 24 h of death (control tissue) or surgical procedures (AAA). GSE47472 with the GPL10558 platform (Illumina HumanHT-12 V4.0 expression beadchip) was obtained from 14 patients with AAA (mean maximum aortic diameter = 62.6 ± 18.0 mm) and 8 control aortic specimens of organ donors. We summarized the demographic characteristics of the 3 datasets (Supplementary Table 1).

### 2.2. Expression Database of the SIRT6-Knockout Mouse Group

The gene expression profile data (GSE178432) with whole-exon microarray analysis for brain samples of the full-body SIRT6-KO and wild-type (WT) mice were selected. There were 8 samples analyzed in the study, of which there were 3 old WT mice (22-26 months old), 2 young WT mice (21 days old), and 3 young SIRT6-KO mice (21 days old). We defined 3 old WT mice and 2 young WT mice as the WT group and defined 3 young SIRT6-KO as the SIRT6-KO group. The commercial platform of gene expression data was GPL619 ([MoEx-1_0-st] Affymetrix Mouse Exon 1.0 ST Array [probe set (exon) version]), and the annotation file for the GPL619 platform was downloaded from NCBI.

### 2.3. Identification of the Differentially Expressed Genes

The GEO database developed a GEO2R web analysis platform (https://www.ncbi.nlm.nih.gov/geo/geo2r/), which enables users to analyze GEO data quickly and conveniently [21, 22]. We performed GEO2R to screen the DEGs in the AAA group compared to the control group and the DEGs in SIRT6-KO mice and young WT mice. The cut-off criteria were logarithmic value  | log_2_FC | >1 and adjusted *P* value < 0.05. ∣Log_2_FC | >1 was defined as the upregulated DEG group, and ∣log_2_FC | <1 was defined as the downregulated DEG group. In addition, we utilized R package “ggpubr” (version 0.4.0) and “ggthemes” (version 4.2.4) to create volcano plot for data visualization. The heat map of hierarchical cluster analysis for the DEGs was performed with the R package “pheatmap” (version 1.0.12), and we selected ward.D2 for the clustering method and Euclidean for the distance method in this study.

The DEGs in both of the human AAA group and SIRT6-KO mouse group were selected for the further analysis, which met the following criteria: (1) logarithmic value  | log2FC | >1 and adjusted *P* value < 0.05 and (2) existing in the SIRT6-KO mouse group and existing in at least 1 or 3 human AAA groups. The Venn diagram that shows the logical relation between datasets of the DEGs was used to visualize the data.

### 2.4. GO and KEGG Enrichment Analyses of DEGs

The online web tool DAVID (https://david.ncifcrf.gov/) for functional annotation bioinformatics microarray analysis was performed to conduct GO and KEGG analyses for both of the AAA-related DEGs and the SIRT6-related DEGs [23], and the analysis results were based on *P* < 0.05 as the selection criteria. Then, we performed GO and KEGG analyses for the DEGs related to both AAA and SIRT6-KO and visualize the GO enrichment data with Sankey dot.

## 3. Results

### 3.1. The Expression of SIRT6 in AAA Patients

The results of GEO2R analysis showed that the expression levels of SIRT6 were downregulated for three groups and upregulated for one group in the three datasets, but none of them satisfied statistical significance (adj. *P* > 0.05) (Table 1). By contrast, SIRT6 was upregulated for the 2 groups in the datasets of GSE57691 (adj. *P* < 0.05); however, the threshold of ∣log_2_FC | >1 was not reached.

### 3.2. The SIRT6-Related Genes Screened from the SIRT6-KO Mice

377 gene probes were downregulated and 298 probes were upregulated in SIRT6-KO mice compared to the WT mice, and the top 20 probes (including the probes for SIRT6) were labeled with the gene symbol in the volcano plot (Figure 1(a)). And we visualized the gene network with a heat map plot (Figure 1(b)), which indicated that the expression of the identified DEGs could correctly distinguish the SIRT6-KO mice and the WT mice. The details with full gene name, gene ID, and gene function of top 10 DEGs (Morc1, Cps1, Kynu, Fmo6, Ttn, Pla2g3, Itgad, Sfpq, Fcrls, and Chrna1) in the SIRT6-KO mice compared to the WT mice are listed in Table 2.

### 3.3. The DEGs Related to Both of SIRT6 and AAA

There were top 5 DEGs (KYNU, NPTX2, SCRG1, GRK5, and RGS5) in both of the human AAA group and SIRT6-KO mouse group (Figure 2), which met the following criteria: (1) logarithmic value  | log_2_FC | >1 and adjusted *P* value < 0.05 and (2) existing in the SIRT6-KO mouse group and existing in at least 3 human AAA groups. The details of the 5 genes are listed in Table 3. There were 43 genes (CPS1, KYNU, FANCD2, LAMA2, ARHGAP15, UPB1, ITGAX, TDO2, FKBP5, ARRDC4, TIAM1, RBM7, PEG3, IGFBP3, IBSP, SGCA, COQ2, MFGE8, SPAG5, NPTX2, OTOA, HYAL1, IER5, FMNL1, SULT1A1, HNRNPC, BTG1, LSP1, TMEM100, WDYHV1, PTPN2, SCRG1, TMPO, TPM2, GABRR1, FAM53B, AIF1, GRK5, FYCO1, SLC26A3, RGS5, AGT, and FAT3) in both of the human AAA group and SIRT6-KO mouse group, which met the following criteria: (1) logarithmic value  | log_2_FC | >1 and adjusted *P* value < 0.05 and (2) existing in the SIRT6-KO mouse group and existing in at least 1 human AAA group.

Among the top 5 DEGs, gene expression of Kynu was significantly downregulated with four gene probes (ID: 4499953, 5302484, 5045128, and 4666160) and the adjusted *P* value was 0.000231, 0.002035, 0.004724, and 0.038934, respectively. Rgs5, Nptx2, Scrg1, and Grk5 were slightly upregulated with at least one gene probe, and the adjusted *P* value was 0.049674, 0.033942, 0.044233, and 0.047621, respectively.

### 3.4. GO and KEGG Analyses of the AAA-Related DEGs and the SIRT6-KO-Related DEGs

Top 25 ontology of the SIRT6-KO-related DEGs showed that several biological processes (BP), cellular components (CC), and molecular functions (MF) were enriched in the tissues of thickness aortic wall biopsies (Figure 3(a)). Among them, the top 3 CC of GO analyses were the cytoplasm (count: 4295), membrane (count: 4445), and nucleus (count: 3758). The top 3 BP of GO analyses were transcription DNA-templated (count: 1263), transport (count: 1211), and positive regulation of transcription from RNA polymerase II promoter (count: 704). The top 3 MF of GO analyses were protein binding (count: 2821), metal ion binding (count: 2241), and nucleotide binding (count: 1320).

In addition, KEGG pathways were enriched in the thickness aortic wall biopsy tissues of AAA patients (Figures 3(b)), and the top 5 pathways were metabolic pathways (*P* value = 1.92*E* − 10), calcium signaling pathway (*P* value = 2.23*E* − 08), ECM-receptor interaction (*P* value = 7.96*E* − 08), focal adhesion (*P* value = 1.83*E* − 07), and small-cell lung cancer (*P* value = 3.56*E* − 07).

GO and KEGG analyses for the 43 DEGs related to both AAA and SIRT6-KO were performed and visualized with the Sankey plot (Figure 3(c)). We found that nine BP (tryptophan catabolic process to acetyl-CoA, tryptophan catabolic process to kynurenine, tryptophan catabolic process, osteoblast differentiation, positive regulation of endothelial cell differentiation, nitrogen compound metabolic process, negative regulation of cell growth, Rac protein signal transduction, and positive regulation of myoblast differentiation), one CC (membrane), and one MF (actin filament binding) were enriched in both of the human AAA group and SIRT6-KO mouse group.

## 4. Discussion

Previous studies showed that SIRT6 reduces DNA damage and improves telomere function and then reduces the senescence of endothelial cells and maintains their ability to proliferate and form tubes in vitro [24]. After knocking out the GATA5 in mouse endothelial cells, a gene related to blood pressure regulation, the GATA5-KO mice developed vascular endothelial dysfunction due to the destruction of normal endothelial signal transduction [25], and it was found that SIRT6 promoted the expression levels of GATA5 [26]. SIRT6 can protect endothelial cell function by regulating the function of endothelial nitric oxide synthase (eNOS) in mice [26, 27]. However, in our study, the gene expression of the NOS gene family (Nos1, Nos2, and Nos3) and GATA gene family (GATA3, GATA5, and GATA6) did not change significantly after knocking out SIRT6. Here, we report on other potential targets on VSMCs regulated by SIRT6 in this study.

In the present study, we analyzed three gene expression microarray datasets of AAA patients and one dataset of SIRT6-KO mice from the GEO database. The results identified 5 DEGs (KYNU, NPTX2, SCRG1, GRK5, and RGS5) in both of the human AAA group and SIRT6-KO mouse group.

The kynurenine pathway is the therapeutic potential enzyme inhibitor against cardiovascular diseases, and it has two major branches, one of which is mediated by KYNU [28]. It was revealed that KYNU is a crucial gene in atheroma plaque development by performing the bioinformatics tools to identify 118 DEGs from the microarray data of GSE43292 [29]. In this study, we also found that KYNU expression was significantly downregulated with four gene probes in the SIRT6-KO mice compared to the WT mice, suggesting that SIRT6 may play an important role in inhibition of cardiovascular diseases (including AAA probably) by regulating the kynurenine pathway.

RGS5, one of the members of the RGS family, was widely expressed along the pericyte-vascular smooth muscle cell axis in central pulp arterioles during tooth restoration [30]. And this suggests that RGS5 is predominantly expressed in VSMCs, and abundance of RGS5 was significantly increased in VSMCs during remodeling collateral arterioles [31]. Downregulation of RGS5 leads to the induction of migration and the activation of GPCR-mediated signaling pathways, which leads to the activation of mitogen-activated protein kinase directly downstream of the receptor stimulus, and ultimately leads to VSMC hypertrophy [32]. But RGS5 overexpression attenuates the angiotensin-induced activation of mitogen-activated protein kinase in SMC of the human aorta [33]. In this study, RGS5 was slightly upregulated after the SIRT6 gene was knockout, suggesting that it is necessary to verify that SIRT6 is a potential treatment target of AAA via inhibition of gene expression of RGS5 in VSMC.

GRK5, a recently cloned member of the G protein-coupled receptor kinase family, has been shown to phosphorylate and participate in the desensitization of angiotensin II- (Ang II-) type 1A (AT1A) receptors, and Ang II (100 nM) upregulated GRK5 mRNA in VSMC [34]. In our study, GRK5 was slightly upregulated after the SIRT6 gene was knockout. GRK5 and RGS5 were included in the regulation of the G protein-coupled receptor protein signaling pathway via GO analysis, suggesting that the pathway regulated by SIRT6 may play a crucial role in AAA.

NPTX2 is a potential target for cognitive dysfunction of Alzheimer's disease and other nervous system disease based on the previous study [35], and it is reported that SCRG1 is involved in cell growth suppression and differentiation during DEX-dependent chondrogenesis [36], but it lacks the evidence of significant association between VSMCs and NPTX2 or SCRG1 yet.

The present study has limitations such as the small sample size and lack of functional and mechanistic validation in VSMCs.

In summary, although SIRT6 mRNA level itself did not change in the tissues of thickness aortic wall biopsies of AAA patients, SIRT6 may play an important role to regulate several signaling pathways with significant association with AAA, suggesting that SIRT6 mRNA upregulation is a protective factor for VSMCs against AAA.

## Figures and Tables

**Figure 1:** (a) Volcano plot of RNA changes between the SIRT6-knockout mice and the WT mice. Note: red: upregulation of gene expression level; green: downregulation of gene expression level. Shades of color indicate the degree of change in the expression. (b) Heat map of DEGs between the SIRT6-knockout mice and the WT mice.

**Figure 2:** Venn diagram of the DEGs in both of the human AAA group and SIRT6-KO mouse group.

**Figure 3:** (a) Top 25 Gene Ontology of the SIRT6-KO-related DEGs. (b) Enrichment dot bubble of top 25 KEGG pathways of the SIRT6-KOrelated DEGs. (c) Sankey plot of GO analysis with 43 DEGs in both of the human AAA group and SIRT6-KO mouse group.

**Table 1:** The expression of SIRT6 in abdominal aortic aneurysm patients.

Gene symbol	Probe ID	Adj. *P* value	*P* value	*t*	*B*	logFC	GEO ID	Groups
SIRT6	ILMN_1654246	8.77*E* − 01	4.86*E* − 01	-0.70263239	-5.950271	−1.21*E* − 01	GSE57691	Large AAA *vs.* control
SIRT6	ILMN_1654246	0.50380533	2.61*E* − 01	-1.143115	-5.620825	-0.16607878	GSE57691	Small AAA *vs.* control
SIRT6	ILMN_1654246	6.45*E* − 01	4.96*E* − 01	0.6904306	-6.39088	0.1707439	GSE47472	AAA *vs.* control
SIRT6	GI_7706709-S	1	1.36*E* − 01	-1.5706757	-5.216965	-0.37320248	GSE7084	AAA *vs.* control

AAA: abdominal aortic aneurysm.

**Table 2:** Top 10 genes of DEGs in the SIRT6-knockout mice compared to the WT mice.

Gene symbol	Gene ID	Official full name	Gene function
Morc1	17450	MORC family CW-type zinc finger 1	This gene encodes the human homolog of mouse morc, and like the mouse protein, it is testis-specific. Mouse studies support a testis-specific function since only male knockout mice are infertile; infertility is the only apparent defect. These studies further support a role for this protein early in spermatogenesis, possibly by affecting entry into apoptosis because the testis from knockout mice shows greatly increased numbers of apoptotic cells

Cps1	227231	Carbamoyl-phosphate synthase 1	The mitochondrial enzyme encoded by this gene catalyzes synthesis of carbamoyl phosphate from ammonia and bicarbonate. This reaction is the first committed step of the urea cycle, which is important in the removal of excess urea from cells. The encoded protein may also represent a core mitochondrial nucleoid protein. Three transcript variants encoding different isoforms have been found for this gene. The shortest isoform may not be localized to the mitochondrion. Mutations in this gene have been associated with carbamoyl phosphate synthetase deficiency, susceptibility to persistent pulmonary hypertension, and susceptibility to venoocclusive disease after bone marrow transplantation

Kynu	70789	Kynureninase	Kynureninase is a pyridoxal-5′-phosphate- (pyridoxal-P-) dependent enzyme that catalyzes the cleavage of L-kynurenine and L-3-hydroxykynurenine into anthranilic and 3-hydroxyanthranilic acids, respectively. Kynureninase is involved in the biosynthesis of NAD cofactors from tryptophan through the kynurenine pathway. Alternative splicing results in multiple transcript variants

Fmo6	226565	Flavin-containing monooxygenase 6	This gene is a pseudogene, and the diseases associated with FMO6P include trimethylaminuria

Ttn	22138	Titin	This gene encodes a large abundant protein of striated muscle. Mutations in this gene are associated with familial hypertrophic cardiomyopathy 9, and autoantibodies to titin are produced in patients with the autoimmune disease scleroderma

Pla2g3	237625	Phospholipase A2 group III	This gene encodes a protein that belongs to the secreted phospholipase A2 family, whose members include the bee venom enzyme. The encoded enzyme functions in lipid metabolism and catalyzes the calcium-dependent hydrolysis of the sn-2 acyl bond of phospholipids to release arachidonic acid and lysophospholipids. This enzyme acts as a negative regulator of ciliogenesis and may play a role in cancer development by stimulating tumor cell growth and angiogenesis. This gene is associated with oxidative stress, and polymorphisms in this gene are linked to risk for Alzheimer's disease

Itgad	381924	Integrin subunit alpha D	This gene belongs to the beta-2 integrin family of membrane glycoproteins, which are composed of noncovalently linked alpha and beta subunits to form a heterodimer. It encodes the alpha subunit of the cell surface heterodimers and is involved in the activation and adhesion functions of leukocytes. The gene is located about 11 kb downstream of the integrin subunit alpha X gene, another member of the integrin family. It is expressed in the tissue and circulating myeloid leukocytes. Alternative splicing results in multiple transcript variants

Sfpq	71514	Splicing factor proline and glutamine rich	The diseases associated with SFPQ include renal cell carcinoma, Xp11-associated and dyslexia

Fcrls	80891	Fc receptor-like S, scavenger receptor	This gene belongs to a class of proteins that resemble Fc receptors. They are preferentially expressed by B lymphocytes. Unlike the classical Fc receptors, there is no strong evidence that suggests that FCRLs bind to the Fc portion of antibodies

Chrna1	11435	Cholinergic receptor nicotinic alpha 1 subunit	The muscle acetylcholine receptor consists of 5 subunits of 4 different types: 2 alpha subunits and 1 each of the beta, gamma, and delta subunits. This gene encodes an alpha subunit that plays a role in acetylcholine binding/channel gating. Alternatively spliced transcript variants encoding different isoforms have been identified

**Table 3:** The details of top 5 DEGs related to both of SIRT6 and AAA.

Gene symbol	Gene ID	Official full name	Gene function
KYNU	70789	Kynureninase	Kynureninase is a pyridoxal-5′-phosphate- (pyridoxal-P-) dependent enzyme that catalyzes the cleavage of L-kynurenine and L-3-hydroxykynurenine into anthranilic and 3-hydroxyanthranilic acids, respectively. Kynureninase is involved in the biosynthesis of NAD cofactors from tryptophan through the kynurenine pathway. Alternative splicing results in multiple transcript variants

NPTX2	4885	Neuronal pentraxin 2	This gene encodes a member of the family of neuronal pentraxins, synaptic proteins that are related to C-reactive protein. This protein is involved in excitatory synapse formation. It also plays a role in clustering of alpha-amino-3-hydroxy-5-methyl-4-isoxazolepropionic acid- (AMPA-) type glutamate receptors at established synapses, resulting in nonapoptotic cell death of dopaminergic nerve cells. Upregulation of this gene in Parkinson disease (PD) tissues suggests that the protein may be involved in the pathology of PD

SCRG1	11341	Stimulator of chondrogenesis 1	Scrapie-responsive gene 1 is associated with neurodegenerative changes observed in transmissible spongiform encephalopathies. It may play a role in host response to prion-associated infections. The scrapie-responsive protein 1 may be partly included in the membrane or secreted by the cells due to its hydrophobic N-terminus. In addition, the encoded protein can interact with bone marrow stromal cell antigen 1 (BST1) to enhance the differentiation potentials of human mesenchymal stem cells during tissue and bone regeneration

GRK5	2869	G protein-coupled receptor kinase 5	This gene encodes a member of the guanine nucleotide-binding protein- (G protein-) coupled receptor kinase subfamily of the Ser/Thr protein kinase family. The protein phosphorylates the activated forms of G protein-coupled receptors thus initiating their deactivation. It has also been shown to play a role in regulating the motility of polymorphonuclear leukocytes (PMNs)

RGS5	8490	Regulator of G protein signaling 5	This gene encodes a member of the regulators of G protein signaling (RGS) family. The RGS proteins are signal transduction molecules which are involved in the regulation of heterotrimeric G proteins by acting as GTPase activators. This gene is a hypoxia-inducible factor-1-dependent, hypoxia-induced gene which is involved in the induction of endothelial apoptosis. This gene is also one of three genes on chromosome 1q contributing to elevated blood pressure. Alternatively spliced transcript variants have been identified

## Data Availability

The data used to support the findings of this study are available from the corresponding author upon request.

## Supplementary Materials

Supplementary Materials Supplementary Table 1: demographic features of 5 RNA expression datasets from microarray analyses of the AAA disease.
